# Anti-Inflammatory and Antibacterial Potential of Qicao Rukang Powder in Bovine Subclinical Mastitis

**DOI:** 10.1155/2021/2148186

**Published:** 2021-08-27

**Authors:** Bereket H. Imam, Ayodele O. Oladejo, Xiaohu Wu, Jie Yang, Xiaoyu Ma, Wenxiang Shen, Jiang Wei, Zuoting Yan, Xuezhi Ding

**Affiliations:** ^1^Key Laboratory of Veterinary Pharmaceutics Discovery, Lanzhou Institute of Husbandry and Pharmaceutical Sciences of Chinese Academy of Agricultural Science, Lanzhou 730050, China; ^2^Department of Veterinary Science, Hamelmalo Agricultural College, Keren 397, Eritrea; ^3^Department of Animal Health Technology, Oyo State College of Agriculture and Technology, Igboora, Nigeria

## Abstract

**Background:**

Subclinical mastitis is one of the most common reproductive diseases in dairy cows. Qicao Rukang powder is a Chinese herbal compound mixture developed to treat subclinical mastitis in dairy cows by clearing heat, tonifying qi, and improving blood and milk circulation. The study aimed to determine the anti-inflammatory and antimicrobial efficacy of Qicao Rukang powder in treating subclinical mastitis in dairy cows at the manufacturer's recommended dose.

**Methods:**

Forty (40) Holstein dairy cows with milk somatic cell count (SCC) ≥ 500,000 cellml^−1^ were randomly assigned to treatment (*n* = 20) and control (*n* = 20) groups. Cows in the treatment group were administered with 150 grams of Qicao Rukang powder orally for five days, while the control group received no treatment. The authors analyzed the milk SCC, milk composition, bacteriological cure rate of the drug, blood serum levels of interleukins (IL-6, IL-1*β*, and IL-8), tumor necrosis factor (TNF-*α*), and interferon gamma (INF-*γ*) quantified by using ELISA kits on day 0 and day 6.

**Results:**

SCC of the treated group reduced very significantly (*P* < 0.001) compared with the control group. Milk fat, protein, and total solids increased significantly (*P* < 0.05) after treatment, whereas lactose and milk urea nitrogen levels showed a nonsubstantial rise. The bacteriological cure percentage of Qicao Rukang powder therapy was 77.8% for *Aeromonas* spp. (14 of 18), 75% for *Pseudomonas* spp. (6 of 8), and 100% for *Acinetobacter* spp. and *Enterococcus* spp. giving 81.8% cured for all isolates (27 of 33). Only 26.7% (8 of 30) of untreated cows recovered spontaneously. Analysis of IL-1*β*, IL-6, and INF-*γ* in the blood serum of the treated group revealed a significant decrease (*P* < 0.01) with nonsignificant rises in TNF-*α* and IL-8 levels.

**Conclusions:**

This research demonstrates that Qicao Rukang powder has potent antibacterial and anti-inflammatory actions, supporting its use as an alternative to conventional treatment for subclinical dairy cow mastitis. However, further investigations will be required to explain the role of the active ingredients and the mechanisms involved in the pharmacological activities of the Qicao Rukang powder.

## 1. Introduction

Dairy cow mastitis is one of the major diseases threatening the development of dairy cattle breeding worldwide [1] and is the inflammation of the mammary gland caused primarily by invading of pathogenic microorganisms [2, 3]. It causes significant economic losses by reducing milk production, profit margins, milk quality, and veterinary costs [4, 5].

Clinical mastitis (CM) and subclinical mastitis (SCM) are the two types based on clinical manifestations. SCM is 15–40 times more common than CM and more challenging to detect. Subclinically infected cows are the primary source of transmission to other healthy cows [6]. A study on the prevalence of subclinical mastitis in dairy cows in eastern China's Gansu Province found that 25.92 percent of cows had subclinical mastitis [7]. Subclinical mastitis has a systemic effect on the reproduction capacity of the infected animal [8]. It can be diagnosed by elevated somatic cell counts, milk production losses, and the presence of inflammatory mediators and bacteria in milk [9]. An increase in milk somatic cell count (SCC) regulated by inflammatory indicators can reflect the damage to the mammary gland. The host reaction to these inflammations varies noticeably in the production of cytokines [10, 11]. Cytokines are one of the immunoregulatory mediators mainly employed to investigate mammary gland immune responses and evaluation of mastitis [12].

Antibiotics and ointments such as penicillin, sulfa, macrolides, tetracycline, and streptomycin have played an essential role in preventing and treating dairy cow mastitis [13]. However, its long-term use is cost correlated, developed drug-resistant bacteria, attributes antibiotic residues via milk to human health hazards, and disrupts the host's symbiotic gut flora [13–15]. Nowadays, researchers are looking for more appropriate and safer natural treatment options for prevention against many diseases, including bovine mastitis worldwide [16]. Chinese herbal component mixtures provide enhanced therapeutic value than chemical and biological agents, which aimed to solve the biosystem as a whole to alter the body's entire immune system and produce long-term results [17]. They also contain a range of nutrients, including polysaccharides and proteins [18].

Qicao Rukang powder is a pharmaceutical product mainly composed of *Astragalus membranaceus* (Fisch.) Bge. Var. mongholicus (Bge.), *Leonurus japonicus* Houtt. (Laur.) S.Y. Hu, and *Vaccaria segetalis* (Neck.) Garcke. Many reports have shown that each component of the Chinese herbal compound mixture exhibits different pharmacological activities; for instance, *Astragalus membranaceus* (root) enhances the body's defense system [19] and possesses anti-inflammatory [20], antioxidant and antihyperglycemic [21, 22], expectorant, diuretic impact, and hepatoprotective actions [23]. *Vaccaria segetalis* (Seed) activates blood circulation, suppresses swelling mastitis and pain, and stimulates milk flow to relieve pains from galactostasis [24]. *Leonurus japonicus* (aerial part) extracts have antibacterial action [25] to regulate menstrual disorders and postdelivery bleeding, as well as to enable blood circulation, diuretics, and edema dispelling [26]. After all, the mechanism for treating subclinical mastitis is not yet documented.

The current study was conducted to investigate the anti-inflammatory and antibacterial efficacy of orally administered Qicao Rukang powder in subclinical mastitis dairy cows for the first time. Changes in somatic cell count (SCC), milk composition, and bacteriological curative percentage were observed from the milk sample. The expressions of proinflammatory cytokines (IL-1*β*, INF-*γ*, TNF-*α*, and IL-6) and chemokine (IL-8) in blood serum was evaluated before and after treatment within the group and between treatment and control groups.

## 2. Materials and Methods

### 2.1. Tested Drug and Reagents

The tested drug, Qicao Rukang powder, was purchased from the manufacturer, Zhengzhou Bairui Animal Pharmaceutical Co., Ltd., with License No. 16067 and GMP certificate no. 16009 (Zhengzhou city, China). The E.Z. N.A Bacterial DNA Kit was bought from Omega Bio-Tek, Norcross, GA. Universal primers forward (27F) and reverse (1492R) were purchased from Beijing Tsingke Biotechnology Co., Ltd. (Beijing, China). Bovine-species-specific (ELISA kits), namely, interleukins (IL-1*β*, IL-6, and IL-8) and tumor necrosis factor (TNF-a), and interferon gamma (INF-γ) were ordered from TSZ Biological Trade Co., Ltd., San Francisco, CA, USA LOT 202009. The Gram stain kit was bought from Beijing solarbio life science and technology Co., Ltd. Others, such as Lanzhou mastitis test (LMT) solution and agarose, were provided by the Lanzhou Institute of Animal Husbandry and Pharmaceutical Sciences. Blood agars were bought from Guangdong Huankai Microbial Sci and Tech. co., ltd., China. Additional materials utilized in these experiments came from approved sources and were of analytical grade.

### 2.2. Experimental Animal Preparation

The research was carried out in the Liaoyuan ranch dairy farm in Gansu Province, China, from May until September 2020. Nearly 1000 Holstein dairy cows were maintained in similar housing, dietary, and managerial circumstances. They were milked by using a rotary milking machine (Ruishengyuan Machinery Assembly Co., Ltd., Hebei, China). A total of 40 apparently healthy lactating cows with an initial age of 3–5 years, 650–800 kg (714 ± 60) body weight, 2–4 parity, and 2–6 months postpartum were registered for the study based on the history of the previous mastitis. The subclinical mastitis was confirmed by the Lanzhou mastitis test.

### 2.3. Subclinical Mastitis Screening Method Test

Before sampling, each animal's quarters were palpated for abnormalities in form, size, edema or udder atrophy, and consistency. Likewise, a quarter of the milk sample was observed for any gross abnormality in milk. Following that, milk samples were screened using People's Republic of China Agricultural Industry Standard NY/T2692-2015, Lanzhou mastitis test (LMT), a rapid diagnosis technology for cows with subclinical mastitis. This rapid field test used an LMT diagnostic solution, in which 5 ml of fresh milk sample was added to a test paddle to mix with 5 mL LMT solution, immediately accompanied by a gentle rotation in the horizontal direction of the mixture. The reaction was visualized within 30 seconds, and the result was scored as “−,” “±,” “+,” “+ +,” and “+ + +” corresponding to *N*, *T*, 1, 2, and 3, representing negative, trace, weakly positive, distinctly positive, and strongly positive results for subclinical mastitis, respectively [27]. Forty (40) dairy cows with at least two quarters showed that the LMT result scored (+) and above was judged as suffering from subclinical mastitis and registered for the study (Figure 1).

### 2.4. Experimental Design, Sampling, and Processing

Based on the results of the LMT screening test, the study animals were randomly divided into two groups: the treatment group (*n* = 20), which received 150 g of Qicao Rukang powder orally for five consecutive days based on the producer's information, and the control group (*n* = 20), which received no treatment. Milk samples were taken from both the treated and nontreated groups on the day (0) before and day (6) following the last experiment. After discarding the first three to four streams of milk, 40 mL of composite milk was collected aseptically into 50 mL sterilized tubes and placed in a cold chain for quick analysis upon transport to the laboratory. In the laboratory, 1 ml of milk was separated into a 2 ml collection tube for bacterial isolation, and the remaining milk was analyzed for composition and somatic cell count. Simultaneously, blood samples were obtained from the same animal's coccygeal (tail) vein on days (0) and (6) while the animal was restrained in the crush. Using one hand holding the tail, fecal material was wiped off the ventral surface of the tail with a swab. The blood was drawn with a vacutainer needle attached to a vacuum blood collection tube (Jiangxi Medical Treatment Co., Ltd.) and transferred to the laboratory in an ice-filled transport cooler. Blood samples were centrifuged at 4°C at 2,700 rpm for 20 minutes in the laboratory, and the serum was extracted and stored at −20°C for further analysis.

### 2.5. Ethics Statement

All the methods involving animals and their welfare were approved by the Institutional Animal Care and Use Committee of Lanzhou Institute of Animal Husbandry and Pharmaceutical Sciences of Chinese Academy of Agricultural Sciences, China (SYXK-2014-0002). Before beginning of sample collection, the owners of all dairy farms engaged in the study were informed and all blood and milk samples were obtained with their permission. Every effort was made to alleviate animal suffering.

### 2.6. Analysis of Milk Constituents and Somatic Cell Count

Milk fat, protein rate, lactose, total solids, milk urea nitrogen, and somatic cell count were measured automatically using a Fossomatic™ 7 cell counter (Foss analytical, Hilleroad, Denmark) following the manufacturer's instructions. In accordance to the Somatic Cell Count (SCC) cutoff for subclinical mastitis diagnosis in China, milk samples with SCC ≥ 500,000 cells ml^−1^ deemed to suffer from subclinical mastitis [28].

### 2.7. Isolation and Bacteriological Analysis of Mastitis Pathogens

The bacteriological examination was carried out in accordance with the National Mastitis Council's guidelines [29]. 10 *µ*l of each fresh milk sample was spread onto a blood agar plate containing 5% defibrinated sheep blood for primary isolation of bacteria. Inverted plates were incubated aerobically at 37°C for 24–48 hours and observed every 24 hours for colony identification. Characterization of bacterial isolates was mainly carried out using the method described by Cowan [30] with some modifications. Bacteria colony count of FO (F zero generation) plates was recorded as follows: extremely dense for single colony counts ≥1000/plate, more dense for 100–1000 colonies/plate, dense for 50–100 colony counts/plate, and scare for 1–50 colonies/plate (Figure 2). To obtain pure colonies, in the subsequent generations (*F*1, *F*2, or *F*3), the representative colonies were again subcultured into new agar plates followed by every time incubation for 18 to 24 h at 37°C. Bacterial colonies were then tentatively categorized based on morphology, Gram stain, and hemolysis patterns. After 48 hours of incubation, plates without bacterial growth are determined if no bacteria growth is seen on the plate. A cow was identified as cured if the pathogen isolated from the pretreatment sample was not separated from the posttreatment samples and if the colony count decreased to scare (1–50 mixed colonies per plate) level after treatment.

Bacterial genomic DNA was extracted from purified colonies using the E.Z.N.A Bacterial DNA Kit (Omega Bio-Tek, Norcross, GA) according to the manufacturer's information. The DNA fragments recovered were checked for concentration using the NanoDrop Technique. The filtered DNA was used for polymerase chain reaction (PCR) amplification. Approximately full-length 16S rRNA genes (1520 bp) were amplified to determine milk sample bacterial community, using the universal primers 27F (5′-AGAGTTTGATCCTGGCTCAG-3′) and 1492R (5′-GGTTACCTTGTTACGACTT-3′). Amplification parameters were as follows: a 5-minute denaturing step at 94°C, followed by 30 cycles of 1 minute at 94°C, annealing 1 minute at 55°C, extension at 72°C for 1 minute, and a final extension at 72°C for 10 minutes; the separated DNA fragments and PCR products were subjected to gel electrophoresis (1% agarose). The purified products submitted to the company for sequencing and the compiled sequences were recognized to the species level by performing a BLAST search against 16S rRNA sequences at the National Center for Biotechnology Information (NCBI, http://www. ncbi.nlm.nih.gov).

### 2.8. Cytokine Quantification Using Enzyme-Linked Immunosorbent Assay (ELISA)

Blood serum levels of tumor necrosis factor (TNF-a), interferon (INF-*γ*), and interleukins (IL-1*β*, IL-6, and IL-8) were determined using commercially available bovine-species-specific ELISA kits (TSZ Biological Trade Co., Ltd., San Francisco, CA, USA LOT 202009) based on the manufacturer's instructions. ELISA tests were assayed in duplicate. An automated plate reader was used to take absorbance readings at 450 nm (ELx800, Bio-Tek Instruments, Winooski, VT). The results were computed by combining the OD sample values with the relevant standard curve and represented as ng/l.

### 2.9. Statistical Analysis

For statistical analysis, GraphPad® Prism 7.00 Software (GraphPad Software, Inc. 7825 Fay Avenue, Suite 230 La Jolla, CA 92037, USA) was used. Some data seemed to be normally distributed, while others appeared to be nonnormal, according to the D'Agostino and Pearson normality test and the Shapiro–Wilk normality test. As a result, for nonnormal data, we used a nonparametric Wilcoxon matched-pairs signed-rank test and a parametric *T* test for normal data. Welch's correction was used for normal data. The Mann–Whitney U test was used for nonparametric data to assess the effect of the tested drug between the control and treatment groups (independent samples). Data are depicted in the bar graph as mean ± SD.

## 3. Results

### 3.1. Milk Somatic Cell Count

#### 3.1.1. Analysis between Paired Samples

In the Qicao Rukang powder-treated group, the number of subclinical mastitis cows with an average milk SCC of 1629 ± 312 *∗* 103 cellsml^−1^ decreased from 20 pretreatments to 3 posttreatments, which gives 85% (17 out of 20) of the cows' SCC restored to the normal level (336 ± 133 *∗* 103 cellsml^−1^). No significant change (1019 ± 230 *∗* 103 cellsml^−1^) was observed in the control group, and only 35% (7 out of 20) of cows spontaneously restored their SCC to normal levels (Figure 3).

#### 3.1.2. Analysis between Independent Groups

The effect of Qicao Rukang powder on SCC of mastitis cows in both the control and treatment groups was evaluated. To generate one independent column for each group, the SCC of the composite milk sample assessed on day six was subtracted from its equivalent pretreatment values on day 0. The Mann–Whitney U test was used, and the results showed a significant difference (*P*=0.0024, *U* = 90).

### 3.2. Effect of Qicao Rukang Powder on Milk Components and Milk Yield

Milk components such as milk fat, protein, and total solids were increased significantly in the Qicao Rukang powder-treated group (Table 1). In comparison, the lactose and milk urea nitrogen percentage increased from 5.8 ± 0.1 to 5.9 ± 0.1 and from13.9 ± 0.6 to 14.4 ± 0.4, respectively. In the control group, no substantial change was observed.

### 3.3. Bacteriological Analysis

Of bacteria isolated from milk samples of cows in the Qicao Rukang powder-treated group, *Aeromonas* spp., 18 of 33 (54.5%), *Pseudomonas* spp., 8 of 33 (24.2%), *Acinetobacter* spp., 4 of 33 (12.1%), and *Enterococcus* spp., 3 of 33 (9.1%), were the primary causative pathogens of subclinical mastitis. For the control group, *Aeromonas* spp., 15 of 30 (50%), *Pseudomonas* spp., 10 of 30 (33.3%), *Acinetobacter* spp., 3 of 30 (10%), and *Enterococcus* spp., 2 of 30 (6.7%), were the isolated causative agents. The range of pathogens causing subclinical mastitis to treatment and control groups is shown in Table 2. After treatment, *Aeromonas* spp. isolates were found to be cured by 77.8% (14 of 18), 75% for *Pseudomonas* spp. (6 of 8), and 100% for *Acinetobacter* spp. and *Enterococcus* spp., giving 81.8% cured for all isolates (27 of 33). Only 26.7% (8 of 30) of untreated cows recovered spontaneously.

### 3.4. Proinflammatory Cytokine and Chemokine Levels

#### 3.4.1. Evaluation between Paired Samples

The trends of changes in IL-8, TNF-*α*, IL-6, IL-1*β*, and INF-*γ* serum concentration from day 0 before to day 6 after treatment were tested using the paired *t* test as shown in Figure 4. The blood serum levels of IL-8 and TNF-*α* showed a similar pattern of change with an insignificant rise (*P* > 0.05) after treatment. However, significant (*P* < 0.05) reduced IL-6, IL-1*β*, and INF- *γ* were detected in serum on day six after treatment compared with the blood serum on day 0 before treatment. At the same time, no substantial change was observed on day six compared to day 0 in the control group.

#### 3.4.2. Between Independent Groups

The unpaired *t* test with Welch's correction for the normal data and Mann–Whitney U test for the nonnormal data were used to compare the anti-inflammatory effects of the Chinese herbal component mixture between the control and treatment groups. In this analysis, the blood serum concentrations of each proinflammatory cytokine (IL-8,TNF,IL-1*β*, IL-6, and INF-*γ*) evaluated at day 6 were subtracted from their correspondent pretreatment values at day 0 to form one independent column for each group. The test revealed an insignificant difference in IL-8 (*t* = 0.9604 df = 35.31, *r*^2^ = 0.02546) and TNF-*α* (*t* = 1.936 df = 37.05,*r*^2^ = 0.09189) but a significant difference for IL-1*β* (*t* = 2.41 df = 31.7, *r*^2^ = 0.1549, *P*=0.0219), IL-6 (*t* = 0.152 = 2.492 df = 34.65, *r*^2^ = 0.152, *P*=0.0176), and INF-*γ* (*U* = 114.5, *P*=0.0199) between control and treatment groups.

## 4. Discussion

Several efforts have been made in China to find a safer natural therapy containing essential active ingredients for treating subclinical mastitis in dairy cows. Puxing Yinyang San (PYS), a compound of herbs, has shown to be effective in preventing and treating subclinical mastitis in dairy cows, with an efficacy rate of 88.89% [31]. In mice and rats, it was demonstrated to have analgesic and anti-inflammatory actions [32].

At the time of this report, there have been no published scientific papers exploring the use of Qicao Rukang powder in the treatment of subclinical mastitis. However, each chemical component of the Chinese herbal compound mixture has been extracted, and a wide range of pharmacological effects was determined. The polysaccharides, saponins, and flavonoids are the main antibacterial bioactive compounds of *Astragalus membranaceus* [33, 34]; others, compounds such as flavonoids, phenolic acids, glucuronic acid, amino acids, and traces of folic acid, have been searched in humans and animals as potential anti-inflammatory, antioxidant, and antihyperglycemic coumpounds [23, 35]. *Leonurus japonicus*, known to contain many chemical constituents, mainly monoterpenoids [36], sesquiterpenoids and steroids [37], and alkaloids and flavonoids [38], which exhibits antibacterial action, has the ability to regulate menstrual disorders, enable blood circulation, diuretics, and edema dispelling [39]. A wide range of chemical compounds is extracted from the seed of *Vaccaria segetalis*, including alkaloids, triterpene saponins, phenolic acid, cyclic peptide, steroids, and flavonoids [40, 41]. These compounds have been determined to activate blood circulation, suppress swelling mastitis and pain, and stimulate milk flow to relieve pain from galactostasis [42].

The current study found that orally administering Qicao Rukang powder to dairy cows with subclinical mastitis for five days eliminated 82.6% (19 isolates out of 23) of the mastitis pathogens. As a result, the milk SCC in the treated cows decreased significantly, the blood serum level of systemic inflammatory mediators reduced, and milk composition increased. In the untreated control group, there was no noticeable difference.

The penetration of pathogenic bacteria into the mammary gland produces toxins, enzymes, and cell wall components that can induce inflammation. The inflammatory process stimulates infiltrations of immune cells from blood to the site of infection, resulting in an elevated milk SCC, thereby increasing systemic proinflammatory cytokines and chemokines [43, 44]. The immune response either destroys the pathogens by phagocytosis or creating reactive oxygen molecules and antimicrobial peptides. In this study, we showed that oral administration of 150 g Qicao Rukang powder for five days in subclinical mastitis cows significantly (*P* < 0.001) reduced milk SCC (Figure 3). The decrease in SCC milk could be because Qicao Rukang powder contains various active ingredients, such as polysaccharides, which have a wide range of biological activities that can boost immunity and help prevent and treat mammary gland diseases [45]. In a relevant search conducted by Jin et al. [46] using extracts of *Tinospora cordifolia*, which contains active ingredients such as alkaloids, polysaccharides, proteins, and phenol, after intramammary infusion of the extracts, the somatic cell count decreased significantly (*P* < 0.05) on day 15 of the treatment period. High SCC in dairy cows is an indication of subclinical mastitis. Low SCC (1.5 × 105 cellsml^−1^) usually implies being free of infection [47].

Subclinical mastitis affects milk's composition and physical and chemical properties [48]. Evaluation of milk components including milk fat, protein, and total solids indicated a significant increase (*P* < 0.05) in the Qicao Rukang powder-treated group when compared to pretreatment values (Table 1). Possible reasons could be that the tested drug contains antioxidants and anti-inflammatory activities that can help maintain rumen microbial balance by reducing potential pathogens. This increased rumen bacteria responsible for increasing total volatile fatty acid (VFA) production but decreased NH3 concentration. As the population increases, more milk or meat is made [49, 50]. Chinese herbal medicine contains bioactive components and many nutrients such as polysaccharides and proteins that could increase milk yield of livestock effectively without toxic side effects and residue [51, 52].

Bacteriological analysis of the present study of milk samples obtained from a commercial dairy farm revealed bacteria, such as *Aeromonas* spp. (52.4%), *Pseudomonas* spp. (28.6%), *Acinetobacter* spp. (11.1%), and *Enterococcus* spp. (7.9%), were the most prevalent causative agent of subclinical mastitis for both treatment and control groups (Table 2). Similar findings of Ozavci et al. [53] showed *Aeromonas* spp. was the most isolated agent from milk samples of dairy cows with subclinical mastitis. Some epidemiological studies indicated a shift in pathogens, from major to minor pathogens, which may play a significant role in the pathogenesis of mastitis [54, 55]. The reason might be due to the change in the management system for dairy cattle industries worldwide and should not be ignored. Posttreatment results obtained in this study showed *Aeromonas* spp. isolates were found to be cured by 77.8% (14 of 18), *Pseudomonas* spp. by 75% (6 of 8), and 100% for *Acinetobacter* and *Enterococcus* spp. Only 26.7% (8 of 30) of untreated cows recovered spontaneously. The total bacterial curative percent was 81.8% (27 of 33) for all isolates after treatment. The nonspecific antimicrobial action was suggested to be due to polysaccharides, saponins, flavonoids, steroids, and other active compounds present in Qicao Rukang powder. The active ingredients of different compound herbs have been determined to exhibit solid antimicrobial action by inhibiting microbial adherence to mucosal or epithelial surfaces, suppressing endotoxin shock, and selective inhibition of microbial growth [56].

The secretion of pro- and anti-inflammatory cytokines is crucial for any immune response. Our research evaluated blood serum levels of TNF-*α*, IL-1*β*, IL-6, INF-*γ*, and IL-8 using the ELISA test which indicated a change in serum level after treatment (Figures 4(a)–4(e)), in which serum concentrations of IL-8 and TNF-*α* showed a nonsignificant rise. In contrast, the levels of IL-1*β*, IL-6, and INF-*γ* were significantly reduced, demonstrating that the active components of the tested Chinese herbal compound mixture have anti-inflammatory properties. In the control group, no apparent changes were observed. Several bioactive compounds such as saponins, alkaloids, terpenes, flavonoids, coumarin, volatile oil, and ketones extracted from different medicinal plants have been reported to be responsible for anti-inflammatory activities [57]. The composite drugs may exert anti-inflammatory effects by inhibiting inflammatory cytokines and mediators, blocking inflammatory signals, or interfering with chemokines [58, 59]. Different authors performed a similar study investigating the concentration of cytokine expressions. They found higher serum levels of IL-1*β* and IL-2, TNF-*α*, IL-6, and IFN-*γ* in subclinical mastitis compared to control cows [60]. Relevant research was conducted to treat subclinical mastitis through the intramammary infusion of unconventional herbal drugs called *Prosopis juliflora* alkaloids. The alkaloids reduced the expression of IL-1, IL-6, IL-8, and IFN-*γ* in milk serum, indicating that they have an excellent anti-inflammatory effect in vivo [61].

Traditional Chinese medicines have been widely used to treat diseases, most of which play a therapeutic role after being metabolized by the gut flora [62]. Heat-clearing Chinese herbs such as *Scutellaria baicalensis, Forsythia suspensa*, and *Radix Isatidis* have been formulated according to the traditional Chinese medicine concept to eliminate internal heat. They are generally used as antibiotics and antipyretic agents and are, therefore, considered effective in treating inflammatory diseases and microbial infections [63, 64]. The research progress of the chemical components and wide range of pharmacological properties with more minor side effects of herbal preparations are studied at home and abroad [65]. The present work analyzed the anti-inflammatory and antimicrobial potentials of Qicao Rukang powder to provide a particular reference for its further research development.

## 5. Conclusions

Current research has shown that the Chinese herbal compound mixture, Qicao Rukang powder, has demonstrated effective anti-inflammatory and antibacterial activity when orally administered to dairy cows with subclinical mastitis at the manufacturer's dose. Treatment efficacy was measured by analyzing somatic cell count (SCC), milk composition, bacteriological cure rate, and the cytokine profile compared to the control group. The main bioactive constituents in Qicao Rukang powder are considered to be polysaccharides, saponins and flavonoids, monoterpenoids, sesquiterpenoids, alkaloids, cyclic peptides, phenolic acid, and steroids, which possess antibacterial and anti-inflammatory actions (literature). However, further investigations are required to explain the role of the active ingredients and the mechanisms involved in the pharmacological activities of the Qicao Rukang powder. The current research provides direct initial information for intending researchers and, thus, potential recommendation of Qicao Rukang powder to dairy farmers as an anti-inflammatory and antimicrobial agent in tackling incessant postpartum mastitis.

## Figures and Tables

**Figure 1:** **LMT** test result: left rear (LR) teat scored as 1“+,” right rear (RR) scored as 2“++” representing for 50 < SCC ≤ 150 *∗* 104 cellsml^−1^ and 150 < SCC ≤ 500 *∗* 104 cellsml^−1^, respectively, and left front (LF) and right front (RF) scored negative “−” with SCC ≤ 50 *∗* 104 cellsml^−1^.

**Figure 2:** Blood agar plates showing *F* zero generations (*F*o) of particular cultured bacteria from milk samples of the same cow on day 0 (a) and day 6 (b) of the control group. (c, d) Grown bacteria from the milk sample of another cow inoculated on day 0 (c) before and day 6 (d) after treatment of the treated group. Plates (a–c) exhibit extremely dense (≥1000 bacteria colony count) and plate (d) shows scare (1–50) colony count. In this interpretation, the treated cow (d) is considered as cured.

**Figure 3:** SCC of the composite milk sample analyzed on day 0 (before) and day six (end of the experiment) for the control (*n* = 20) and treated groups (*n* = 20). Unlike the SCC of the control group (*P* > 0.05), the SCC of the treated group decreased significantly (*P* < 0.001) when compared to its pretreatment values (paired *t* test). Data were expressed as mean ± SD.

**Figure 4:** (a–e) Blood serum concentration of IL-8 (a), TNF (b), IL-1*β* (c), IL-6 (d), and INF-*γ* (e) in the control and treatment groups. The level of IL-8 and TNF-*α* was nonsignificantly increased at *P* > 0.05 and IL-1*β*, IL-6, and INF-*γ* was significantly reduced at *P* < 0.01 after treatment (day 6) when compared to their pretreatment values (day 0). In the control group, no substantial difference was observed between the values of day 0 and day 6. Data were evaluated by the paired *t* test (IL-8, IL-1*β*, IL-6, and INF-*γ*) and Wilcoxon signed-rank test (TNF-*α*). Bar graphs indicate the mean ± SD.

**Table 1:** Averages observed and standard error of the mean (mean ± SEM) of five milk constituents and milk yield of the treatment group (*n* = 20) and control group (*n* = 20).

Milk components and milk yield	Qicao Rukang powder treatment group		Control group	
	RX 0	RX 6	Day 0	Day 6
Milk fat	3.9 ± 0.12	4.8 ± 0.2^*∗*^	3.9 ± 0.12	4 ± 0.14
Protein rate	3.3 ± 0.1	3.5 ± 0.1^*∗*^	3.1 ± 0.1	3 ± 0.1
Lactose	5.8 ± 0.1	5.9 ± 0.1	6 ± 0.1	5.8 ± 0.1
Total solids	12.9 ± 0.2	14 ± 0.3^*∗*^	12.4 ± 0.2	11.2 ± 0.2
Milk urea nitrogen	13.9 ± 0.6	14.4 ± 0.4	13.2 ± 0.6	13.4 ± 0.4
Milk yield	32.7 ± 1.39	35.12 ± 1.18	35.44 ± 1.73	35.3 ± 1.1

Day 0 (before) and day 6 (after) treatment are represented by RX 0 and RX 6, respectively, corresponding to the control (nontreated) group's day 0 and day 6 sampling dates. At *P* > 0.05, values marked with an asterisk (^*∗*^) indicate a significant increase.

**Table 2:** Isolated pathogens that cause subclinical mastitis in both groups at pretreatment and the curative percentage of the Qicao Rukang powder (TCM) evaluated after treatment (*n* = 20), in comparison to untreated mastitis cows (*n* = 20).

Bacteria spp.	Qicao Rukang powder treatment group			Control group		
	Time of sampling		% cured	Time of sampling		% cured
	RX0	RX6		Day 0	Day 6	
*Aeromonas* spp.	18	4	77.8	15	10	33.3
*Pseudomonas* spp.	8	2	75	10	7	30
*Acinetobacter* spp.	4	0	100	3	3	0
*Enterococcus* spp.	3	0	100	2	2	0
Total	33	6	81.8	30	22	26.7

RX 0 and RX 6 symbolize day 0 (before) and day 6 (after) treatment, respectively, and correspond to the day 0 and day 6 sampling periods for the control (nontreated) group.

## Data Availability

All data are available within the manuscript to access without restriction.
